# A Concerted HIF-1α/MT1-MMP Signalling Axis Regulates the Expression of the 3BP2 Adaptor Protein in Hypoxic Mesenchymal Stromal Cells

**DOI:** 10.1371/journal.pone.0021511

**Published:** 2011-06-27

**Authors:** Sébastien Proulx-Bonneau, Amel Guezguez, Borhane Annabi

**Affiliations:** Laboratoire d'Oncologie Moléculaire, Centre de recherche BIOMED, Département de Chimie, Université du Québec à Montréal, Quebec, Canada; University of South Florida, United States of America

## Abstract

Increased plasticity, migratory and immunosuppressive abilities characterize mesenchymal stromal cells (MSC) which enable them to be active participants in the development of hypoxic solid tumours. Our understanding of the oncogenic adaptation of MSC to hypoxia however lacks the identification and characterization of specific biomarkers. In this study, we assessed the hypoxic regulation of 3BP2/SH3BP2 (Abl SH3-binding protein 2), an immune response adaptor/scaffold protein which regulates leukocyte differentiation and motility. Gene silencing of 3BP2 abrogated MSC migration in response to hypoxic cues and generation of MSC stably expressing the transcription factor hypoxia inducible factor 1alpha (HIF-1α) resulted in increased endogenous 3BP2 expression as well as cell migration. Analysis of the 3BP2 promoter sequence revealed only one potential HIF-1α binding site within the human but none in the murine sequence. An alternate early signalling cascade that regulated 3BP2 expression was found to involve membrane type-1 matrix metalloproteinase (MT1-MMP) transcriptional regulation which gene silencing abrogated 3BP2 expression in response to hypoxia. Collectively, we provide evidence for a concerted HIF-1α/MT1-MMP signalling axis that explains the induction of adaptor protein 3BP2 and which may link protein binding partners together and stimulate oncogenic MSC migration. These mechanistic observations support the potential for malignant transformation of MSC within hypoxic tumour stroma and may contribute to evasion of the immune system by a tumour.

## Introduction

Mesenchymal stromal cells (MSC), most commonly isolated from the bone marrow, are a population of pluripotent adult stem cells that can differentiate into many mesenchymal phenotypes [1], [2]. In fact, recruitment of MSC by experimental vascularizing tumours resulted in the incorporation of MSC within the tumor architecture [3], [4] which, combined to intrinsic immunomodulatory mechanisms, implies that they must also respond to tumour-derived growth factor cues [5], [6]. Importantly, the microenvironment and stroma required for the evolution and progression of solid tumours has been investigated over the past few years, and MSC, which are the progenitors of stromal cells and fibroblasts, have been found to interact with cancer cells [7]. Consequently, their potential contribution to tumour development implies that MSC must adapt to the low oxygen environment and nutrient deprivation that characterizes hypoxic tumours.

Homing of MSC to tumours is thought to be among the earliest phenomenon of MSC-cancer interactions, as was recently reported in a mouse model where injected human MSC could be found preferentially migrating to implanted human melanoma tumours [3]. Subsequently, studies have shown MSC homing to tumours and even to sites of metastasis [8]. Furthermore, cotransplantation of MSC with melanoma cells in mice enhanced tumour engraftment and growth [9]. These data are in agreement with observations that vascular progenitors derived from bone marrow stromal cells are recruited by tumours both *in vivo* and *in vitro* [5]. The sum of this evidence, in line with their increased ability to migrate under an atmosphere of low oxygen [10], suggests that MSC are active participants in the development of hypoxic solid tumours.

In order to survive within the stressful hypoxic tumour microenvironment, cells have developed a coordinated set of responses orchestrating their adaptation to hypoxia. The outcomes of such cellular responses to hypoxia are aggressive disease, resistance to therapy, and decreased patient survival [11]. A critical mediator of the hypoxic response is the transcription factor hypoxia inducible factor 1 (HIF-1) which upregulates expression of proteins that promote angiogenesis, anaerobic metabolism, and many other survival pathways [12]. Regulation of HIF-1α, a component of the HIF-1 heterodimer, occurs at multiple levels including translation, degradation, and transcriptional activation, and serves as a testimony to the central role of HIF-1. Unfortunately, the roles played by many of the individual molecular components which merge these different signals remain undefined. Adaptor proteins which link protein binding partners together and stimulate formation of signalling complexes [13] play an important role in the regulation of multiple intracellular signalling pathways that regulate cell mobilization, oncogenesis, metabolic and immunologic adaptative capacities. Among these, the adaptor protein 3BP2 was originally identified as a protein that interacts with the Src homology (SH) 3 domain of the protein tyrosine kinase Abl [14]. 3BP2 is predominantly expressed in hematopoietic/lymphoid tissues and its SH2 domain has been shown to associate *in vitro* with Syk, ZAP70, linker for activation of T cells, Grb2, phospholipase Cγ1, and cbl from activated T cell lysates [15]. Whether any 3BP2 functions are linked to MSC's oncogenic transformation activities, including extracellular matrix (ECM) degradation and directed cell migration, is currently unknown.

While most of the matrix metalloproteinases (MMP) are secreted, MT1-MMP is a membrane-associated MMP regulated by hypoxia [10] and, aside from its well-known role in the activation of proMMP-2 and intrinsic proteolytic activity towards ECM molecules, drives MSC mobilization [16], [17]. More importantly, its cytoplasmic domain was recently shown to link adaptor protein p130Cas [18] and Src-mediated events through the phosphorylation of its intracellular domain [19]. In light of such scaffolds taking place in MT1-MMP cellular signalling, MT1-MMP functions associated with platelet-mediated calcium mobilization [20], regulation of cell death/survival bioswitch [21], [22], and regulation of proinflammatory signalling [23], [24] have been reported. Given that hypoxia is a condition that promotes oncogenic processes, we questioned whether any HIF-1α/3BP2/MT1-MMP signalling axis may contribute to the hypoxic adaptation of MSC.

## Materials and Methods

### Materials

Sodium dodecylsulfate (SDS) and bovine serum albumin (BSA) were purchased from Sigma (Oakville, ON). Cell culture media were obtained from Life Technologies (Burlington, ON). Electrophoresis reagents were purchased from Bio-Rad (Mississauga, ON). The enhanced chemiluminescence (ECL) reagents, protein G- and A-coupled sepharose were from Amersham Pharmacia Biotech (Baie d'Urfé, QC). Micro bicinchoninic acid protein assay reagents were from Pierce (Rockford, IL). The polyclonal antibodies were purchased and generated against the MT1-MMP catalytic domain (Chemicon), the MT1-MMP cytoplasmic domain (Abcam), 3BP2 (Abcam) and GAPDH (Advanced Immunochemicals).

### Cell cultures and experimental hypoxic conditions

This study was approved by the “Comité Institutionnel des Risques Biologiques” through the delivery of a written certificate (#10-CIRB-53.3.5). Bone marrow-derived mesenchymal stromal cells (MSC) were isolated from the whole femur and tibia bone marrow of C57BL/6 female mice; cells were cultured and characterized by flow cytometry as previously described [25]. cDNA construct generation and transduction of the MSC-HIF-1α was performed and extensively described previously [26]. Hypoxic culture conditions were attained by incubation of confluent cells in an anaerobic box for up to 48 hours [26]. The oxygen was maintained at 1% by a compact gas oxygen controller Proox model 110 (Reming Bioinstruments Co., Redfield, NY) with a residual gas mixture composed of 94% N_2_ and 5% CO_2_. Re-oxygenation was kept at its minimum through rapid processing (less than 10 seconds) of the hypoxic cells for total RNA and protein extractions. Serum starvation is classically performed by culturing the cells in high glucose Dulbecco's modified Eagle's medium (DMEM; GibcoBRL) and 100 units/ml Penicillin/Streptomycin, and from which the 10% inactivated fetal bovine serum (iFBS) (Hyclone Laboratories, Logan, UT) was removed.

### Immunoblotting procedures

Cells from MSC or MSC-HIF-1α were lysed and proteins were separated by SDS–polyacrylamide gel electrophoresis (PAGE). After electrophoresis, proteins were electrotransferred to polyvinylidene difluoride membranes and immunoreactive material was visualized by enhanced chemiluminescence as described previously [26].

### Cell survival and migration assays

MSC lysed in Apo-Alert lysis buffer (Clontech, Palo Alto, CA) were assessed for apoptotic cell death by the fluorometric caspase-3 activity as previously described by us [25]. Upon treatment, floating cells were aspirated and removed. Adherent MSC or MSC-HIF-1α were then trypsinized and viability evaluated by Trypan blue exclusion staining. Majority of the cells were found viable and seeding of 10^5^ viable cells was performed on 0.15% gelatin/PBS precoated Transwells (Corning/Costar; Acton, MA; 8-µm pore size) assembled in 24-well Boyden chambers which were filled with 600 µl of serum-free media. Cell migration was allowed to proceed for 6–24 hours at 37°C in 5% CO_2_. The migration was quantified by analyzing at least ten random fields per filter for each independent experiment as described previously [26].

### Total RNA isolation, cDNA synthesis and real-time quantitative RT-PCR

Total RNA was extracted from MSC monolayers using TRIzol reagent (Life Technologies, Gaithersburg, MD). For cDNA synthesis, 1 µg of total RNA was reverse-transcribed into cDNA using a high capacity cDNA reverse transcription kit (Applied Biosystems, Foster City, CA). cDNA was stored at −80°C prior to PCR. Gene expression was quantified by real-time quantitative PCR using iQ SYBR Green Supermix (BIO-RAD, Hercules, CA). DNA amplification was carried out using an Icycler iQ5 (BIO-RAD, Hercules, CA) and product detection was performed by measuring binding of the fluorescent dye SYBR Green I to double-stranded DNA. The following primer sets were provided by QIAGEN (Valencia, CA): HIF-1α (Mm_Hif1a_1_SG QT01039542), 3BP2 (Mm_Sh3bp2_1_SG QT00100464), MT1-MMP (Mm_Mmp14_1_SG QT01064308), VEGF (Mm_Vegfa_1_SG QT00100464), β-Actin (Mm_Actb_2_SG QT01136772). The relative quantities of target gene mRNA against an internal control, β-Actin RNA, were measured by following a ΔC_T_ method employing an amplification plot (fluorescence signal *vs.* cycle number). The difference (ΔC_T_) between the mean values in the triplicate samples of target gene and those of β-Actin RNA were calculated by iQ5 Optical System Software version 2.0 (BIO-RAD, Hercules, CA) and the relative quantified value (RQV) was expressed as 2^−ΔC^_T_.

### Transfection method and RNA interference

MSC were transiently transfected with 20 nM siRNA against HIF-1α (Mm_Hif1a_1 HP siRNA, SI00193011), MT1-MMP (Mm_Mmp14_2 HP siRNA, SI00177800), 3BP2 (Mm_Sh3bp2_4 HP siRNA, SI00204218) or scrambled sequences (AllStar Negative Control siRNA, 1027281) using Lipofectamine 2000 transfection reagent (Invitrogen, CA). HIF-1α-, 3BP2- and MT1-MMP-specific gene knockdown was evaluated by qRT-PCR as described above. Small interfering RNA and mismatch siRNA were synthesized by QIAGEN and annealed to form duplexes.

### Statistical data analysis

Data are representative of three or more independent experiments. Statistical significance was assessed using Student's unpaired *t*-test Probability values of less than 0.05 were considered significant and an asterisk identifies such significance in the figures.

## Results

### Hypoxic culture conditions upregulate 3BP2 gene expression

MSC were serum-starved and cultured under hypoxic conditions as described in the Methods section. Total RNA was then extracted and qRT-PCR performed. We found that hypoxia significantly induced HIF-1α transcript levels (Fig. 1, black bars) in agreement with previous reports [26], [27]. Moreover, 3BP2, VEGF and MT1-MMP gene expression were also induced. These observations suggest that 3BP2 transcriptional regulation occurs in MSC upon low oxygen tension culture conditions. Whether HIF-1α was specifically involved in direct 3BP2 gene regulation was next explored through sequence promoter analysis. An approximate 1,000 bp sequence upstream of the ATG coding sequence of the respective human (NCBI source NC_000004.11 and located on human chromosome 4 at location 2,821,348–2,822,347) and murine (NCBI source NC_000071.5 and located on mouse chromosome 5 at location 3,488,412–3,489,415) 3BP2 gene promoter sequence was analyzed for HIF putative transcription factor binding sites with PROMO 3.0 (http://alggen.lsi.upc.es/) using version 8.3 of the TRANSFAC database. Only one core consensus sequence of the hypoxia responsive elements (A_G)CGT(G_C)C (−28/−23) was found in the human. None was found in the murine sequence analyzed (data not shown). This suggests that alternate players may be involved in the molecular cascade that leads to 3BP2 expression through HIF.

**Figure 1:** Hypoxic culture conditions upregulate 3BP2 gene expression. Subconfluent MSC were serum-starved and cultured under normoxic (5% CO_2_ and 95% air; white box) or hypoxic (1% O_2_, 5% CO_2_ and 94% N_2_; black box) conditions for 18 hours. Total RNA was extracted and quantitative reverse transcription-polymerase chain reaction was performed in order to assess 3BP2, HIF-1α, VEGF and MT1-MMP gene expression levels. Values are means of two independent experiments, each performed in triplicates. Bars, ±SD.

### Gene silencing of HIF-1α antagonizes the effects of hypoxia on 3BP2 gene and protein expression

In order to assess the potential contribution of HIF-1α to 3BP2 gene and protein expression regulation under hypoxic culture conditions, gene silencing strategies were employed to specifically and efficiently down-regulate HIF-1α gene expression in MSC (Fig. 2A, left panel). Such knockdown did not trigger apoptotic cell death as assessed through caspase-3 activity (Fig. 2A, right panel). Mock (scrambled mismatched siRNA) or siHIF-1α-transfected MSC were generated by transient transfection as described in the Methods section. Cells were then cultured under hypoxic culture conditions for 48 hours, total RNA was extracted and qRT-PCR was used to assess 3BP2 gene expression. While 3BP2 gene expression was induced by hypoxia in Mock-transfected cells, we found that its gene expression was efficiently reduced in siHIF-1α-transfected MSC (Fig. 2B). 3BP2 protein expression was also assessed in Mock- and in siHIF-1α-transfected cells that were subsequently cultured under hypoxic conditions (Fig. 2C). While 3BP2 protein expression was increased by hypoxia with a maximal plateau expression occurring between 24 and 48 hours in Mock cells, those cells where HIF-1α gene expression was abrogated (>78%) were unable to increase 3BP2 (Fig. 2D). The relevance of HIF-1α was also assessed on the transcriptional regulation of vascular endothelial growth factor (VEGF) and of membrane type-1 matrix metalloproteinase (MT1-MMP), two important players in MSC survival and mobilization processes [10], [16], [17]. Both the VEGF and MT1-MMP transcript levels were found induced by hypoxic culture conditions, while such regulation was abrogated in siHIF-1α-transfected MSC (data not shown). Consequently, expression of HIF-1α is required for 3BP2 gene and protein regulation upon hypoxia.

**Figure 2:** Gene silencing of HIF-1α antagonizes the effects of hypoxia on 3BP2 gene and protein expression. MSC were transiently transfected with scrambled sequences (Mock, white bars, open circles) or HIF-1α siRNA (black bars, closed circles) as described in the Methods section. Cells were then cultured under normoxic or hypoxic culture conditions as described in the legend of Fig. 1. (A) Apoptotic cell death was assessed using the fluorometric caspase-3 activity assay as described in the Methods section. Concanavalin-A-treated MSC (grey bars) was used as a positive inducer of caspase-3 [16]. Total RNA was extracted, and qRT PCR was used to assess 3BP2 and HIF-1α transcript levels. (B) 3BP2 gene expression was assessed by qRT-PCR in Mock-transfected and in siHIF-1α-transfected cells that were subsequently cultured under hypoxic conditions. (C) Mesenchymal stromal cells were transiently transfected with scrambled sequences or HIF-1α siRNA as described in the Methods section. Cells were then cultured under normoxic or hypoxic culture conditions, cell lysates were isolated, western blotting and immunodetection was performed with anti-3BP2 and anti-GAPDH antibodies. A representative blot is shown out of two. (D) Scanning densitometry was used to assess protein expression described in panel C, and the ratio of 3BP2/GAPDH expression was represented. Values in (A) and (B) are means of two independent experiments, each performed in triplicates (*p<0.05 versus mock control in (A) or mock at time = 0 hr hypoxia in (B)); Bars, ±SD.

### 3BP2 silencing abrogates MSC migration in response to hypoxic culture conditions

In order to assess any 3BP2-mediated cellular impact, cell migration was monitored under normoxic or hypoxic culture conditions. 3BP2 gene silencing was performed (Fig. 3A, upper and middle panels) and found not to trigger apoptotic cell death (Fig. 3A, lower panel). While 3BP2 silencing did not affect basal MSC migration under normoxic conditions (Fig. 3B), cells in which 3BP2 expression was abrogated were unable to respond to hypoxic cues (Fig. 3C, black bars). This suggests that 3BP2 is required for the hypoxic adaptation of MSC that is reflected by an increase in MSC migration.

**Figure 3:** 3BP2 silencing abrogates MSC migration in response to hypoxic culture conditions. MSC were transiently transfected with scrambled sequences or with 3BP2 siRNA as described in the Methods section. (A) Immunoblotting of 3BP2 protein expression was evaluated in cell lysates from Mock (white bars) and siRNA (black bars) experiments. Total RNA was extracted, and qRT-PCR was used to assess 3BP2 gene expression knockdown efficiency. Apoptotic cell death was assessed by the fluorometric caspase-3 activity as described in the Methods section. (B) Cells were harvested and seeded onto Boyden chambers using gelatin-coated filters to assess cell migration under normoxic or hypoxic culture conditions. (C) Cell migration was quantified as described in the Methods section and expressed as x-fold induction over Mock-transfected cells. Values of cell migration are means of three independent experiments (*p<0.05 versus normoxic mock); Bars, ±SD.

### Constitutive expression of an oxygen-dependent degradation domain HIF-1a mutant triggers 3BP2 gene and protein expression

Recently, experimental evidence has shown that upregulation of HIF-1α plays a pivotal role in hypoxia-induced MSC mobilization, possibly acting via its downstream genes VEGF and SDF-1α [28]. To date, no demonstration of the direct role of HIF-1α overexpression itself was performed. In order to recreate the hypoxic culture conditions that trigger HIF-1α expression in MSC, we generated a deletion mutant of HIF-1α (HIF-1α ΔODD) which causes constitutive expression of HIF-1α, and stably transfected MSC with such construct as described in the Methods section. We found that MSC constitutively and stably expressing HIF-1α ΔODD (MSC-HIF-1α) exhibited an increased intrinsic ability to migrate (Fig. 4A). Such increased migratory potential has been documented previously by us [10], [26] and, although speculative, may potentially involve autocrine regulation through hypoxia-regulated growth factor expression. This may provide efficient mobilization and adaptive behaviour of MSC to oxygen deprived environment. When cell lysates and total RNA were extracted from MSC or MSC-HIF-1α, we found that 3BP2 protein (Fig. 4B) and gene (Fig. 4C) expression were significantly increased in MSC-HIF-1α cells. Noteworthy, 3BP2 gene silencing abrogated MSC-HIF-1α migration to levels equivalent to basal MSC migration (Fig. 4D). This observation confirms that 3BP2 expression is among the mediators involved in the response to hypoxic cues and downstream of HIF-1α signaling.

**Figure 4:** Stable expression of HIF-1α increases 3BP2 basal expression and MSC migration. MSC stably expressing a ΔODD HIF-1α mutant (MSC-HIF) were generated as described in the Methods section. (A) Basal migration of MSC and MSC-HIF was performed as described in the Methods section. Values of cell migration are means of three independent experiments (*p<0.05 versus normoxic MSC). (B) Cell lysates were isolated, western blotting and immunodetection was performed with anti-3BP2 and anti-GAPDH antibodies as described in the Methods section. (C) Total RNA was extracted, and qRT-PCR was used to assess 3BP2 gene expression. (D) Cell migration was quantified as described in the Methods section in Mock- (white bars) and si3BP2- (black bars) transfected MSC or MSC-HIF-1α. Values of cell migration are means of three independent experiments (*p<0.05 versus normoxic mock MSC or MSC-HIF); Bars, ±SD.

### MT1-MMP is a prerequisite for hypoxia-mediated expression of 3BP2 in MSC

Classical roles for MT1-MMP are those involved in directed ECM degradation and subsequent cell migration [29]. New alternate roles highlight MT1-MMP as a signalling molecule since its intracellular cytoplasmic domain has been shown to trigger RhoA and Erk transduction pathways [30], [31]. Moreover, increases in MT1-MMP expression correlated with increased MSC migration in response to hypoxia [10]. Since siHIF-1α abrogated both 3BP2 (Fig. 2) and MT1-MMP (not shown) expression in response to hypoxia, we tested whether a signalling axis might regulate crosstalk between MT1-MMP and 3BP2. We first used gene silencing strategies to down-regulate MT1-MMP gene expression and to assess its specific contribution to 3BP2 gene regulation under hypoxic culture conditions. MSC were transiently transfected with scrambled sequences (Mock) or with MT1-MMP siRNA as described in the Methods section. Cells were then cultured under normoxic or hypoxic culture conditions, total RNA was extracted and qRT-PCR was used to assess MT1-MMP and HIF-1α gene expression. We found that MT1-MMP gene expression was significantly reduced in siMT1-MMP transfected cells while HIF-1α gene expression remained unaffected (Fig. 5A). 3BP2 gene expression was then assessed in Mock-transfected and in siMT1-MMP-transfected MSC in response to hypoxic culture conditions. We found that 3BP2 gene expression was induced by in Mock-transfected cells reaching a plateau at 12 hours of hypoxia, while such induction was abrogated in siMT1-MMP-transfected cells (Fig. 5B). 3BP2 protein expression data were also analyzed and support those of the gene expression regulation of 3BP2 in that siMT1-MMP-transfected MSC did not exhibit increased 3BP2 expression due to hypoxia (Fig. 5C). Consequently, expression of MT1-MMP is a prerequisite for 3BP2 transcriptional regulation upon hypoxia.

**Figure 5:** Gene silencing of MT1-MMP antagonizes the effects of hypoxia on 3BP2 gene expression. MSC were transiently transfected with scrambled sequences (Mock, white bars) or MT1-MMP siRNA (black bars) as described in the Methods section. Cells were then cultured under normoxic or hypoxic culture conditions. (A) Immunoblotting of MT1-MMP protein expression was evaluated in cell lysates from siRNA experiments. Total RNA was extracted, and qRT-PCR was used to assess 3BP2, HIF-1α and MT1-MMP. Apoptotic cell death was assessed using the fluorometric caspase-3 activity assay as described in the Methods section. (B) 3BP2 and HIF-1α gene expression were assessed by qRT-PCR in Mock-transfected (open circles) and in siMT1-MMP-transfected (closed circles) cells that were subsequently cultured under hypoxic conditions. (C) MSC were transiently transfected with either scrambled sequences or MT1-MMP siRNA as described in the Methods section. Cells were then cultured under normoxic or hypoxic culture conditions, cell lysates were isolated, western blotting and immunodetection were performed with anti-3BP2 and anti-GAPDH antibodies. Values in (A) and (B) are means of two independent experiments, each performed in triplicates (*p<0.05 versus mock control in (A) or mock at time = 0 hr hypoxia in (B)); Bars, ±SD.

### MT1-MMP overexpression upregulates 3BP2 gene and protein expression

To test whether MT1-MMP-mediated signalling was involved in the regulation of 3BP2 expression, we short-circuited hypoxia-mediated signalling by directly overexpressing either a full-length wild-type (Wt) recombinant MT1-MMP or its cytoplasmic-truncated form (Δ-cyto) in MSC. Total RNA was thereafter extracted and 3BP2 gene expression assessed by qRT-PCR and compared to Mock-transfected MSC. 3BP2 gene expression was increased in Wt-MT1-MMP-transfected MSC but not in cells that overexpressed the Δ-cyto-MT1-MMP (Fig. 6A). Expression of both recombinant proteins, which retained their extracellular catalytic domain intact, led to functional activation of proMMP-2 at the cell surface as assessed by zymography of the respective conditioned media (Fig. 6B). Transfection efficiency was further assessed by measuring expression of the individual MT1-MMP recombinant forms. Full length and Δ-cyto-MT1-MMP forms were detected when membranes were probed with anti-MT1-MMP generated against the catalytic domain (Fig. 6C), while only the full length MT1-MMP was detected when using the anti-MT1-MMP cytoplasmic domain antibody (Fig. 6C). Using the anti-3BP2 protein expression further confirmed the signalling axis that exists between cell surface MT1-MMP and intracellular induction of 3BP2, as only the Wt form of MT1-MMP led to increased protein levels of 3BP2 (Fig. 6C).

**Figure 6:** 3BP2 induction requires MT1-MMP cytoplasmic domain-mediated signalling. (A) MSC were transiently transfected with pcDNA3.1 (Mock, white bars), a plasmid encoding full length MT1-MMP (Wt, black bars), or a plasmid encoding for a cytoplasmic domain-deleted form of MT1-MMP (Δ-cyto, grey bars). Cells were then cultured under normoxic culture conditions, total RNA was extracted, and qRT-PCR was used to assess 3BP2 gene expression. (B) Gelatin zymography of the conditioned media was used to demonstrate efficient cell surface targeting of the respective Wt and Δ-cyto MT1-MMP recombinant proteins and subsequent ability to retain extracellular catalytic functions and to activate the secreted latent proMMP-2 into active MMP-2. (C) Cell lysates were isolated, western blotting and immunodetection was performed with antibodies recognizing the MT1-MMP catalytic or cytoplasmic domain, anti-3BP2 and anti-GAPDH as described in the Methods section. Values are means of two independent experiments, each performed in triplicates (*p<0.05 versus Wt-MT1-MMP control); Bars, ±SD.

## Discussion

Molecular markers associated with MSC are thought to characterize the brain tumour-initiating cells involved in the development of hypoxic solid tumours such as glioblastomas [32], the most common and aggressive primary brain cancer [33]. It is also believed that a subset of primary glioblastomas derive from transformed stem cells possessing MSC-like properties and retaining partial phenotypic aspects of the MSC nature within the tumours' hypoxic environment [32]. Accordingly, exogenously delivered human MSC were found to localize to human gliomas after intravascular delivery [4]. While VEGF-A was demonstrated to contribute to glioma-induced migration of human MSC [34], this raises the possibility that endogenous MSC may further be recruited into hypoxic gliomas during tumorigenesis and may contribute to the physiological growth of brain tumours *in situ*. More recently, MSC implanted directly within the central nervous system (CNS) to treat experimental autoimmune encephalomyelitis were found to produce local pathology of yet unknown consequences as reflected by the formation of cellular masses within brain parenchyma [35]. Caution therefore arises as of future MSC transplantations within inflamed CNS that characterize neurodegenerative and tumor conditions [36]. Nevertheless, these adaptive cellular conditions have significant pathological implications towards hypoxic solid tumour development. In fact, brain tumour-derived cells which are under hypoxic stress develop an adaptive response that includes an increased rate of glycolysis and angiogenesis or undergo cell death by promoting apoptosis and/or necrosis [37]. The metabolic flexibility that enables MSC to survive under conditions characterized by hypoxia was recently shown to involve a microsomal glucose-6-phosphate transporter [26], a protein not only regulating intracellular glucose cycling but also involved in the regulation of cell survival and chemotaxis through ATP-dependent calcium flux [20], [21], [38].

While MSC are usually cultured under normoxic conditions (21% oxygen), their *in vivo* (patho)physiological “niches” have a much lower oxygen tension. Because of their plasticity, stem cells are particularly sensitive to their environments, and oxygen tension therefore becomes one developmentally important stimulus in stem cell biology as it will play a role in the intricate balance between cellular proliferation and commitment towards differentiation [39], [40]. Under hypoxic conditions, the major transcription factor affecting gene regulation in stem cells is HIF-1 [41]. This transcription factor in turn upregulates expression of several genes involved in angiogenesis, such as bFGF, VEGF, and the VEGF receptors Flk-1 and Flt-1, as well as components of the plasminogen system including the urokinase receptor, and the inhibition of plasminogen activator 1 [41], [42]. Other transcription factors activated by hypoxia include early growth response-1 (Egr-1), which regulates MT1-MMP transcription [43], [44]. Interestingly, MSC isolated from Egr-1^−/−^ mice abrogated MT1-MMP functions in cell survival [25]. In the present study, we show that gene silencing of HIF-1α suppressed MT1-MMP as well as 3BP2 gene induction by hypoxia. Prior silencing of MT1-MMP gene expression also abrogated 3BP2 gene expression by hypoxia. This is suggestive of a cascade of molecular events triggered by HIF, and leading to MT1-MMP-mediated upregulation and possible recruitment of 3BP2 to the plasma membrane that may, in part, explain increased MSC migration. Interestingly, Egr-1 was recently shown to regulate HIF-1α gene expression during hypoxia [45]. While MT1-MMP was shown to trigger the expression of VEGF, which is also a target gene product of HIF-1 and may possibly contribute to an autocrine regulation of increased cell migration [46], [47], we propose that MT1-MMP-mediated regulation of 3BP2 expression may be a key modulator in the proteolytic and cell migratory oncogenic and immunomodulatory responses of MSC under hypoxic conditions.

3BP2 is an adaptor/scaffold protein thought to regulate immune receptor-mediated signal transduction [48], [49], and that takes part in various cellular functions such as apoptosis [48] cell differentiation [50], several signalling pathways [51], reorganization of actin cytoskeleton, cell motility and cell adhesion [50]. Most of the above-mentioned functions are also commonly shared by MT1-MMP in angiogenic processes [52]. Interestingly, 3BP2 silencing is also associated with impaired activation of multiple signalling events downstream of RANK, including actin reorganization, Src, ERK, and JNK phosphorylation, and up-regulation of osteoclastogenic factors [50]. Given the absence of predicted HIF-1α binding sequence within the 3BP2 gene promoter, one may consequently hypothesize alternate signal transduction triggers to be involved in MSC adaptation upon low oxygen environment. In fact, our data confirm that hypoxia-mediated induction of 3BP2 requires a concerted MT1-MMP and HIF-1α signalling. Among the possible chronological events taking place in this HIF-1α/MT1-MMP/3BP2 signalling axis, one can envision a recruitment and binding of 3BP2 at the membrane. Preliminary data arising from immunoprecipitation experiments performed in cells transfected with Wt-or Δ-cyto-MT1-MMP cDNA suggest direct binding of 3BP2 to the cytoplasmic domain of MT1-MMP (not shown). While recruitment of adaptor proteins such as p130Cas and the kinase activity of Src [18], [19] to MT1-MMP suggest that such scaffolds already take place in MT1-MMP-mediated cellular signalling, further studies will be required to better understand the (patho)physiological impact of such dynamic.

Finally, studies have indicated the ability of stem cell populations, including MSC, to inhibit or downregulate immune responses *in vitro* and *in vivo* [53]. MSC have recently been reported to inhibit naive and memory antigen-specific T cells [54]. The immunosuppressive qualities of MSC, which may facilitate evasion of the immune system by a tumour, may in part involve major histocompatibility complex (MHC) class I. Interestingly, phenotypic characterization of MSC by flow cytometry showed expression of MHC class I alloantigens, but failed to elicit T cell proliferative responses due to active suppressive mechanisms [55]. Recently, shedding of the tumour cell surface MHC class I chain-related molecule A by MT1-MMP, a membrane bound matrix metalloproteinase, was demonstrated to regulate sensitivity of tumour cells to NK cell killing, a process which may add to tumour immune evasion and contribute to tumour progression [56]. Such cell surface proteolytic activity of MT1-MMP was also shown in MSC to contribute to cleavage of CD44, another cell adhesion molecule expressed at the cell surface of MSC, and to promote cell migration [31], [57].

MSC present a promising tool for cell therapy as proven effective in pre-clinical studies. In fact, they are currently being tested in US FDA-approved clinical trials for myocardial infarction, stroke, meniscus injury, limb ischemia, graft-versus-host disease and autoimmune disorders [58]. Clinical trials for MSC injection into the CNS to treat traumatic brain injury and stroke are also currently ongoing. Whether hypoxia/ischemia alteration of MSC may influence endogeneous or exogenously transplanted MSC biodistribution fate remains however to be better investigated. Intravenous infusion of MSC was found to reduce brain damage after transient global cerebral ischemia *in vivo* [59]. These neuroprotective features of MSC are likely to occur through some paracrine regulation mechanisms [60]. In support to the MSC paracrine recruitment, MSC transplantation provided trophic support to an ischemia/reperfusion injured liver model by stimulating regeneration [61]. Therapeutic efficacy through MSC mobilization was also demonstrated in a hindlimb ischemia model [62].

Hypoxia is a tissue-specific condition that can promote oncogenic processes. Indeed, in the bone marrow, the hypoxic environment is important for maintaining the stemness, cell cycle, survival and metabolism of MSC and HSC [63]. Moreover, the low oxygen tension is thought to protect the genomic integrity of stem cell populations by limiting the production of reactive oxygen species by the mitochondrial respiration [64]. However, countless evidences provide a role for hypoxia in the mobilization and migration of MSC to the peripheral blood [28] and to tumors [65], [66]. In tumoral context, hypoxia might promote oncogenic progression because of the heterotypic interactions within the tumor stroma. Indeed, hypoxic cancer cells secrete various cytokines, such as IL-6, VEGF, PDGF and FGF, that attract and promote MSC proliferation and differentiation into tumor-supporting cells [67], [68]. The complex nature of the hypoxic tumor microenvironment makes it pro-oncogenic for MSC, as opposed to the hypoxic niche of the bone marrow, which preserves their integrity and function.

In conclusion, our study provides unexpected original molecular evidence linking the adaptor protein 3BP2 to oncogenic transformation contribution of MSC in response to hypoxia. A schematic representation is shown to summarize the possible signalling mechanism that is triggered upon MSC hypoxic cues and that could possibly lead to 3BP2 recruitment to MT1-MMP and to MSC migration (Fig. 7). Furthermore, we document a new molecular signalling axis driven by the intracellular domain of MT1-MMP in concert with signalling requiring HIF-1α, and which adds to the new roles of MT1-MMP as recently described in energy-dependent regulation through non-proteolytic mechanisms [69]. The sum of this evidence supports, in part, the oncogenic and immunomodulatory adaptive mechanisms that could eventually be targeted in MSC that contribute to hypoxic tumour development.

**Figure 7:** Putative mechanisms involved in 3BP2 response to hypoxia and recruitment by MT1-MMP. Scheme summarizing the mechanisms involved in 3BP2 response to hypoxia and potential recruitment by MT1-MMP. Hypoxia induces HIF-1α, which then upregulates MT1-MMP gene transcription, MT1-MMP synthesis and targeting to the plasma membrane. The intracellular domain of MT1-MMP is mandatory to signal potential 3BP2 recruitment and to trigger both cell migration and extracellular matrix (ECM) degradation. proMMP-2, latent form of matrix metalloproteinase-2; MMP-2, active form of matrix metalloproteinase-2; TIMP-2; tissue inhibitor of MMP-2.
